# The Association between the Parents' Knowledge of Carbohydrate Counting and the Glycaemic Control of the Children with Type 1 Diabetes

This article has been retracted.

**DOI:** 10.1155/2018/1036214

**Published:** 2018-06-19

**Authors:** Priyanga Ranasinghe, Vidarsha Rajini Senadeera, Rashmi Senarathna, Uththara Sapurnika, Vindhya Ramanayake, Ranil Jayawardena

**Affiliations:** ^1^Faculty of Medicine, University of Colombo, Colombo, Sri Lanka; ^2^Institute of Health and Biomedical Innovation, Queensland University of Technology, Brisbane, Australia

## Abstract

**Background:**

Medical nutritional therapy is an important component of type 1 diabetes (T1D) care in children and carbohydrate counting is one such method. We aimed to evaluate the knowledge of carbohydrate counting among parents of children with T1D from Sri Lanka and study its association with the child's glycaemic control.

**Methods:**

A descriptive cross-sectional study was conducted among parents of children with T1D. HbA1c measurement was used to assess glycaemic control. Knowledge of parent regarding carbohydrate counting was assessed based on a 24-hour dietary recall. Carbohydrate counting knowledge was defined using ratio of carbohydrate content estimated by parents to actual carbohydrate content calculated by researchers (Total, Breakfast, Lunch, Dinner, and Snacks). Ratios obtained were also divided into three groups, underestimation (<0.9), accurate estimation (0.9-1.1), and overestimation (>1.1). A multivariate regression analysis was performed to determine contribution of carbohydrate counting accuracy to glycaemic control (HbA1c).

**Results:**

Sample size was 181 and mean age of the parents was 38.8±5.9 years. Mean duration of diabetes in the children was 3.7±2.6 years and mean HbA_1_c level was 8.3±0.9%. On average, parents estimates of carbohydrate count for the total meal were 0.88±0.27 (88%) (range 0.38-1.47) of the actual carbohydrate count. Only 30.5% (n=55) of parents were grouped in the “accurate” estimation category for the total carbohydrate count. Parents of children with diabetes for ≤3 years estimated total carbohydrate count more accurately than the counterparts (p<0.05). Mean HbA1c value of those who “underestimated” was significantly higher than those with “accurate” estimation. In the multivariate analysis accuracy of carbohydrate estimation was associated with a lower HbA1c (*β* = −0.36; p=0.03).

**Conclusions:**

Overall knowledge of carbohydrate counting among parents was inadequate. Better knowledge was associated with improved glycaemic control in children and lower incidence of hypoglycaemic episodes. An inverse association was observed between knowledge and duration of diabetes.

## 1. Background

Diabetes mellitus is a chronic noncommunicable metabolic disease characterized by hyperglycemia which occurs due to the relative or absolute deficiency of insulin [1]. Type 1 diabetes (T1D) also known as immune-mediated diabetes, accounts for only 5–10% of those with diabetes [1]. T1D results from a T cell-mediated autoimmune destruction of the *β*-cells of the pancreas over many years, leading to insulin deficiency [1]. The symptoms arise only when 70–90% of *β*-cells have been destroyed; however the extent of *β*-cells destruction varies with age; those who are older at onset tend to have more *β*-cells than young children and loss of 40% of *β*-cells can be sufficient to induce symptoms in a 20-year-old person [2]. The disease usually presents early in life and it is one of the most common chronic diseases of childhood [3]. Peaks in presentation occur between 5 and 7 years of age and at or near puberty [4]. Globally, the incidence and prevalence of T1D vary between countries and regions, being most common in Finland and other Scandinavian countries [5]. Recent studies have shown a steady increase in the prevalence of T1D [1]. The economic burden associated with T1D is likely to be considerable, since the disease presents during childhood or adolescence. It is estimated that each year T1D results in medical costs and lost income of about $14.4 billion in the US [6].

Insulin treatment together with regular blood glucose monitoring is the main treatment strategy for T1D. Medical nutritional therapy is also an important component of T1D care in children [7]. It aims to provide sufficient and appropriate energy as well as macro- and micronutrients for optimal growth, development, and glycaemic control [7]. Carbohydrate counting is one such method which allows the adjustment of prandial insulin dose according to the carbohydrate intake in T1D patients [8]. Standard carbohydrate content of food items is documented and is made available to the patients, which enables them to calculate the carbohydrate amounts in each meal and adjust the insulin doses required to preserve postprandial blood glucose within normal limits [9]. This allows more freedom to the growing child or the adolescent with T1D, by offering more flexibility with their diets [10]. Studies have shown that carbohydrate counting improves glycaemic control in children with T1D [11].

To date most studies on carbohydrate counting have been conducted in western countries. The South Asian diet shows a great deal of variety when compared with the western diet; it is high in carbohydrates,* trans*-fats, and saturated fat [12]. Comparative studies have reported a higher overall caloric intake, as well as a greater percentage of carbohydrate content in a typical South Asian meal, compared with a standard European meal [13]. Therefore carbohydrate counting is likely to be more difficult and complex in the South Asian context. Sri Lanka is a South Asian country with a population of nearly 21 million. Dietary patterns in Sri Lanka are similar to elsewhere in the region and typically have a high carbohydrate content [14]. Hence, it is likely that Sri Lankan parents find carbohydrate counting more challenging, which in turn possibly leads to poor glycaemic control in the children. The present study aims to evaluate the knowledge of carbohydrate counting among parents of children with T1D from Sri Lanka and study its association with the child's glycaemic control and other sociodemographic parameters.

## 2. Methods

### 2.1. Study Population and Sampling

This descriptive cross-sectional study was conducted at the Lady Ridgeway Hospital for Children, Colombo, Sri Lanka. The hospital has a bed strength of over 900 and it is considered to be one of the largest children's hospitals in the world [15]. In addition, children with T1D throughout the country are referred to its clinics from other hospitals and the patients belong to many ethnic groups and diverse socioeconomic backgrounds enabling analysis of different factors that would affect the knowledge of carbohydrate counting. The study was approved by the Ethics Review Committee, Faculty of Medicine, University of Colombo, Sri Lanka, and Institutional Review Committee of the Lady Ridgeway Hospital for Children, Colombo, Sri Lanka. Written informed consent was obtained from all participants prior to recruitment to the study.

The sample size required to calculate a difference of HbA1c 0.5%, between those with good and poor knowledge (SD–1.15, *α*–0.05, and *β*–80%), was 168. A nonresponse rate of 10% was assumed. Hence one hundred and ninety parents of children with T1D satisfying the inclusion and exclusion criteria were invited for the study. For inclusion the child should be diagnosed with T1D at least 6 months before recruitment to the study (in order for the parents to familiarize with carbohydrate counting and for the treatment to be optimized) and treated with multiple daily injections of insulin and use carbohydrate counting in meal planning. Furthermore, the parent had to be the person who counted carbohydrates at home. Children having other concurrent endocrine diseases or disorders interfering with nutritional management were excluded from the study. The clinics are held once per week and on each day those satisfying the inclusion/exclusion criteria were determined and a list of eligible participants was prepared. Subsequently the first patient was selected randomly from this list and thereafter every other patient was invited for the study.

### 2.2. Study Instrument and Data Collection

Data collection was carried out by trained Research Assistants. An interviewer-administered questionnaire was used for collection of sociodemographic and disease related data. The questionnaire evaluated sociodemographic (age and gender of parent/child, level of education of parent, and occupation) and disease related factors (duration of disease, insulin injection frequency and dose, number of hypoglycaemic episodes in past month, and presence of diabetes related complications). HbA1c measurement was used for the assessment of glycaemic control. Knowledge of the parent regarding carbohydrate counting was assessed based on a 24-hour dietary recall of the child's diet by the parent. Initially the parent was asked to recall the previous day's meal taken by the child from 6.00 am to 6.00 am the next day. The meals were separated into Breakfast, Lunch, Dinner, and Snacks. Subsequently the parents were asked to count carbohydrates for each meal based on the dietary recall. Household kitchen measures and two-dimensional food models were used to assist the parents to determine the portion size.

### 2.3. Definitions and Data Analysis

The data collectors used the food item standard carbohydrate content guideline available at the hospital to calculate the actual carbohydrate content of each of the four meals separately. The total carbohydrate content was taken as the aggregate of these four values. The accuracy of these calculations were verified by a single Clinical Nutritionist (RJ) with experience in Sri Lankan dietary patterns and their composition, prior to analysis. A single Clinical Nutrition was utilized in order to minimize interobserver variations. Hypoglycaemic events were defined clinically, as the presence of symptoms related to hypoglycaemia that disappear following treatment with oral or parenteral glucose [16]. Carbohydrate counting knowledge was defined using the ratio of carbohydrate content estimated by parents to the actual carbohydrate content calculated by the researchers. This was done separately for each of the four meals and for the total carbohydrate content. Thus, five ratios were obtained using this method (Breakfast, Lunch, Dinner, Snacks, and Total).

For comparison the ratios obtained were also divided into three groups, underestimation (<0.9), accurate estimation (0.9-1.1), and overestimation (>1.1). This grouping was done separately for the total value and ratios of each meal (Breakfast, Lunch, Dinner, and Snacks). An average Sri Lankan meal consists of 100g of carbohydrates, and previous studies have shown that a carbohydrate counting variation of >10g is associated with glycaemic impairment [14, 17]. Hence, for this analysis, accuracy was defined by estimates within 10% of calculated actual intake (total ratio between 0.9 and 1.1). Furthermore, for analysis purposes the duration of diabetes was divided into two equal groups (≤ 3 years and >3 years); HbA1c levels were grouped as ≤7.50%, 7.51–8.50%, and >8.50% to reflect good, adequate, and poor glycaemic control, respectively, while the participants were grouped based on age as ≤35 years, 36-40 years, and >40 years.

A multivariate regression analysis was performed to determine the contributions of carbohydrate counting accuracy to glycaemic control (HbA1c), adjusting for child's age, parent's age, parent's level of education, and duration of diabetes. Data were analyzed using SPSS version 14 (SPSS Inc., Chicago, IL, USA). Descriptive data are presented as percentages or as mean±SD. Significance of associations was tested using Chi square for categorical variables and Student's t-test or ANOVA for continuous variables. In all analyses a p value ≤ 0.05 was considered statistically significant.

## 3. Results

### 3.1. Sociodemographic Characteristics

Sample size was 181 (response rate was 95.3%) (parent to child ratio 1:1). Majority of the parents were mothers (78.5%, n=142), while 68.5% (n=124) of the children were females. Most of the children were in the 6-10 years' (45.3%, n=82) and 11-15 years' (49.2%, n=89) age categories. The mean age of the parents and children was 38.8±5.9 years (range 23-52 years) and 10.2±2.4 years (range 2-15 years), respectively. Majority of parents were educated up to the level of secondary education (Grades 6-11) (56.4%, n=102), while 9.9% (n=18) have completed tertiary education. Majority of the parents were housewives (64.6%, n=117).

The mean duration of diabetes in the children was 3.7±2.6 years (range 7 months–12 years). Mean HbA_1_c level was 8.3±0.9% and HbA_1_c levels ranged from 5.4 to 10.6%, with only 19.9% (n=36) of the study population achieving an HbA1c value of <7.5%. The mean morning, evening, and night insulin doses were 10.6±6.2 IU, 4.3±4.6 IU, and 6.8±6.1 IU, respectively, while the mean total insulin dose was 21.6±11.3 IU. Majority of the children used insulin three times per day (60.2%, n=109). None of the children had renal complications due to diabetes, although 5% (n=9) had been diagnosed with visual complications. Number of hypoglycemic episodes in the past month ranged from 0 to 3 episodes, while the majority (74.6%, n=135) did not have any episodes; 20.4% (n=37) had only one episode.

### 3.2. Carbohydrate Counting and Sociodemographic Factors

On average, parents estimates of carbohydrate count for the total meal was 0.88±0.27 (88%) (range 0.38-1.47) of the actual carbohydrate count. The ratio values were most accurate for Lunch (1.00±0.53 [range 0.33-4.00]), followed by Breakfast (0.96±0.43 [range 0.33-2.00]) and Dinner (0.88±0.39 [range 0.13-2.00]). Least accuracy was observed for estimation of carbohydrate count in Snacks (1.22±0.58 [range 0.50-3.33]). In the categorical analysis only 30.5% (n=55) of parents were grouped in the “accurate” estimation category for the total carbohydrate count, while “underestimation” (44.2%, n=80) was the most common category. Percentages of parents in the “accurate” estimation category for Breakfast, Lunch, Dinner, and Snacks were 29.8% (n=53), 35.9% (n=65), 29.8% (n=53), and 22.1% (n=40), respectively.

Parental estimate of total carbohydrate count was more accurate in fathers (0.97±-0.18) than in mothers (0.86±0.29) (p=0.014). However, no significant difference in the carbohydrate count between mothers and fathers was noted in the individual meals (Breakfast, Lunch, Dinner, and Snacks) (Table 1). We did not observe a significant association between carbohydrate count ratio and parental age (Table 1). No association between carbohydrate count and age was also observed in the categorical analysis (underestimation/accurate estimation/overestimation) (Table 2). When considering the level of education, the ratio of total carbohydrate count was significantly more accurate in those with secondary education (Grade 6-11) than in those with tertiary education; this was also independently observed for ratios obtained for Breakfast and Snacks (Table 1). Majority of parents (43.6%, n=79) varied between under- and overestimation for individual meals; 16.6% accurately estimated all meals (n=30); the balance, 39.7% (n=72), either consistently underestimated or overestimated all the meals.

### 3.3. Carbohydrate Counting and Diabetes

Parents of children with diabetes for ≤3 years estimated the total carbohydrate count more accurately than those with duration >3 years (Table 1) (p=0.042). However, this difference was not independently observed for individual meals (Breakfast, Lunch, Dinner, and Snacks). Similarly, in the categorical analysis, those with “accurate” estimation of the carbohydrate count (Total, Breakfast, and Snacks only) had a lower mean duration of diabetes in comparison to those with “underestimation” and “overestimation” (Table 2). The total carbohydrate count ratio was significantly more accurate in parents of children with and HbA1c level ≤ 7.5% than in those with HbA1c > 8.5% (Table 1). Furthermore, this was also independently observed in Dinner carbohydrate count ratio. The mean HbA1c value of those who “underestimated” it was significantly higher than those with “accurate” estimation (Total, Lunch, and Dinner) (Table 2). Furthermore, it was also noted that parents of children who had no hypoglycaemic episodes during the past month had estimated total carbohydrate count more precisely than those of children experiencing hypoglycaemia (Table 1). This was also observed independently for carbohydrate counting of Dinner and Snacks (Table 1). In the multivariate analysis adjusting for child's age and duration of diabetes, accuracy of carbohydrate estimation was associated with a lower HbA1c (*β* = −0.361 [95% CI −0.57 to −0.15]; p=0.03). The overall model was significant (p=0.01) and accuracy of carbohydrate counting explained 5% of the variance in HbA1c in the model.

## 4. Discussion

To our knowledge this is the first study from South Asia evaluating the association between carbohydrate counting knowledge among parent's and the glycaemic control of children with T1D. Our results show that better knowledge of carbohydrate counting among parents was associated with improved glycaemic control in children with T1D (measured by HbA1c). We were also able to identify that better knowledge was associated with lower incidence of hypoglycaemia. In addition mothers and parents with higher levels of education had lesser knowledge in comparison to their counterparts. The duration of diabetes in children was inversely associated with knowledge.

In the present study population less than 1/3^rd^ had good knowledge about carbohydrate counting, with nearly 69.5% either over/underestimating the carbohydrate values in the meal. Previous studies from western developed countries such as USA and Ireland have demonstrated better carbohydrate counting knowledge among parents [11, 18]. The observed difference could be due to the better socioeconomic status and health literacy in these countries, in comparison to Sri Lanka. However, this argument is not fully supported by the observation that lower education was associated with better knowledge in the present population. The typical South Asian diet is high in carbohydrates,* trans*-fats, and saturated fat [12]. It can sometimes be difficult to count the amount of carbohydrates in the complex South Asian meals and lack of accurate nutritional data with regard to commonly consumed local meals further compounds the situation [19]. This could be one of the reasons for the observation of high rates of over- and underestimation of the carbohydrate values in the present population. Furthermore, the carbohydrate estimation for Snacks was the least accurate (27.6%), with the widest variations in measurement. This also supports the above finding, since Snacks in South Asia can often be complex in composition and varied in quantity, making standardization and quantification difficult for accurate carbohydrate estimation. It is important to note that other available studies have not compared the knowledge of the parents with regard to the specific meal, unlike in the present study. Although we observed a significant difference in the accuracy levels with regard to estimation of carbohydrates in Snacks, we did not see a major difference between the other three meals (Breakfast, Lunch, and Dinner).

Our results show that better parental knowledge of carbohydrate counting was associated with improved glycaemic control, while underestimation of carbohydrates was associated with a higher HbA1c. Several individual studies have also noted similar observations among children [11, 17, 20]. However this has been contradicted elsewhere, where studies have reported superior glycaemic outcomes from other interventions in comparison to carbohydrate counting in children [21]. A recent systematic review and meta-analysis of interventional studies comparing carbohydrate counting with general/alternate dietary advice reported a 0.64% reduction in HbA1c in the carbohydrate counting group compared to controls, mainly in adults [22]. However, the authors reported significant heterogeneity between studies and there was only one study involving children [22]. Absence of carefully designed controlled interventional studies in children is a barrier to decide on the effectiveness of carbohydrate counting on glycaemic control [8]. We also note the presence of suboptimal glycaemic control in the present study population (mean HbA1c, 8.3%), with only 19.8% (n=36) of the study population achieving an HbA1c value of <7.5%. Inadequate knowledge regarding carbohydrate counting and meal planning could be one of the contributory causes for the poor glycaemic control observed.

The results of our study also demonstrate that better knowledge of carbohydrate counting can help to reduce hypoglycaemic episodes among the children. For individuals with T1D, hypoglycemia is the most common acute side effect of insulin therapy and serves as one of the major barriers to optimal glycaemic control, presenting a significant challenge for children and their parents in attempting to achieve optimal management of blood glucose levels [23]. Hence, when adopting carbohydrate counting for meal planning and glycaemic control in children, it is very important to educate and train parents regarding the proper technique of carbohydrate counting, in order to minimize errors and reduce the risk of inadvertent hypoglycaemia. Furthermore, our results also indicate an inverse association between carbohydrate counting knowledge in parents and the duration of diabetes. Similar results have been observed when children were involved in carbohydrate counting, highlighting the need for age-appropriate diabetes education as the child grows older [24]. However, in instances such as the present study, where adults were involved in carbohydrate counting, improvement in accuracy would have been expected with increasing duration, owing to better experience. This highlights the need for continuous education and training even among adults. It seems indispensable for both parent and children to continuously practice carbohydrate counting under the guidance of health care professionals and appropriate educational materials to maintain the accuracy of estimation over time [25].

There are several limitations which are noted in the present study. Dietary recall was used as the method to assess the knowledge of parents regarding carbohydrate counting. Reliance on memory may limit the validity of diet recalls in assessing the actual carbohydrate intake in children [26]. Hence, other studies have adopted food models for knowledge assessment. However, in the Sri Lankan context the 24-hour dietary recall was selected as being most appropriate, because the ethnic diversity and associated variations in food habits restrict the use of standard food models, which would unduly bias the knowledge assessment. Furthermore, we did not assess other factors which are known to affect HbA1c, such as carbohydrate quality and other disease related factors, such as number of DKA (Diabetic Ketoacidosis) episodes. In addition, hypoglycaemia was defined clinically, due to the lack of home glucometers for most families to define hypoglycaemia by blood glucose values.

## 5. Conclusions

The overall knowledge of carbohydrate counting among parents was inadequate. Better knowledge was associated with improved glycaemic control in the children and lower incidence of hypoglycaemic episodes. We also observed an inverse association between knowledge and duration of diabetes. Our sample included children with relatively poorly controlled T1D and parents were mostly from a middle level socioeconomic background; hence our findings need to be further strengthened by confirmation in more diverse populations.

## Figures and Tables

**Table 1:** Knowledge of carbohydrate counting expressed with a ratio and its associations.

	Carbohydrate Count (Mean ± SD) (Ratio between estimated value and actual value)				
	Total	Breakfast	Lunch	Dinner	Snacks
Parental Status					
Mother (n=142, 78.5%)	0.86±0.29^*∗*^	0.96±0.46	1.00±0.58	0.85±0.40	1.19±0.58
Father (n=39, 21.5%)	0.97±0.18^*∗*^	0.97±0.33	1.00±0.25	0.93±0.35	1.29±0.62

Parental Age					
≤ 35 years (n=40, 22.1%)	0.92±0.26	0.91±0.54	0.94±0.28	0.87±0.33	1.19±0.61
36-40 years (n=80, 44.2%)	0.82±0.27	0.86±0.35	0.89±0.46	0.86±0.48	1.15±0.61
> 40 years (n=61, 33.7%)	0.92±0.25	0.93±0.44	0.89±0.67	0.92±0.30	1.14±0.49

Level of Education					
Secondary Education (Grades 6-11) (n=102, 56.4%)	0.92±0.24^*∗∗*^	0.94±0.38^¥^	1.03±0.44	0.91±0.41	1.02±0.68^≠^
Advance Level (Grades 12-13) (n=61, 33.7%)	0.87±0.29	0.96±0.48	0.94±0.66	0.87±0.39	1.00±0.25^†^
Tertiary Education (n=18, 9.9%)	0.75±0.24^*∗∗*^	1.21±0.54^¥^	1.03±0.51	0.77±0.24	0.71±0.19^≠†^

Duration of Diabetes					
≤ 3 years (n=90, 49.7%)	0.93±0.26^∞^	0.96±0.39	0.95±0.42	0.86±0.41	1.15±0.47
> 3 years (n=91, 50.3%)	0.82±0.27^∞^	0.96±0.47	1.05±0.61	0.91±0.37	1.27±0.66

HbA1c Level (%)					
≤ 7.50 (n=36, 19.9%)	0.92±0.14^≠^	0.96±0.42	0.96±0.30^*∗∗*^	0.90±0.37	1.01±0.12
7.51 – 8.50 (n=59, 32.6%)	0.85±0.18	0.93±0.41	0.93±0.30	0.91±0.34	1.05±0.43
> 8.50 (n=76, 42.0%)	0.79±0.16^≠^	0.93±0.33	0.78±0.19^*∗∗*^	0.85±0.40	1.15±0.51

Hypoglycaemic episodes (last month)					
None (n=135, 74.6%)	0.96±0.28^≠^	0.97±0.44	1.04±0.28^≠^	0.89±0.39	1.00±0.34
≥ 1 episode (n=46, 25.4%)	0.82±0.21^≠^	0.94±0.41	0.85±0.30^≠^	0.87±0.39	1.30±0.30

^*∗*^p-0.014, ^*∗∗*^p-0.002, ^*¥*^p-0.03,  ^≠†^p<0.001, and ^*∞*^p-0.042. Values in the same column with the same superscript are significantly different from each other; significance of associations was tested using Student's t-test or ANNOVA.

**Table 2:** Knowledge of carbohydrate counting expressed with categories and its associations.

	Mean ± SD				
	Total	Breakfast	Lunch	Dinner	Snacks
Parental age					
Under estimation	38.92±5.44	38.97±5.71	38.23±5.35	38.92±5.51	40.93±4.48
Accurate estimation	39.00±7.08	39.69±5.79	38.80±6.55	39.80±6.81	38.83±5.95
Over estimation	38.44±5.59	36.63±6.20	39.66±5.48	37.00±4.75	37.18±7.28

Duration of Diabetes (years)					
Under estimation	4.77±1.83^*∗*^	4.26±3.02^*∗*^	3.98±3.04	3.78±2.85	4.26±3.14^*∗*^
Accurate estimation	2.96±1.85^*∗*†^	3.27±2.25^*∗*†^	3.36±2.49	3.55±2.23	3.11±1.31^*∗*†^
Over estimation	4.48±1.85^†^	4.56±2.37^†^	3.84±2.02	3.89±3.09	4.33±1.17^†^

HbA1c Level (%)					
Under estimation	8.40±0.98^*∗*^	8.30±1.05	8.86±0.98^*∗*^	8.52±0.84^*∗*^	8.17±1.24
Accurate estimation	8.06±0.98^*∗*†^	8.39±0.94	8.11±0.89^*∗*^	8.16±0.92^*∗*^	8.16±1.21
Over estimation	8.53±0.90^†^	8.25±1.03	8.26±0.93	8.22±1.07	8.37±0.82

^*∗*^p<0.01; ^†^p<0.05. Values in the same column with the same superscript are significantly different from each other.

## Data Availability

The datasets used and/or analyzed during the current study are available from the corresponding author on reasonable request.

## Abbreviations

ANOVA: Analysis of variance
DKA: Diabetic Ketoacidosis
HbA1c: Glycosylated haemoglobin
IU: International units
SD: Standard deviation
T1D: Type 1 diabetes
US: United States.
